The article "Effect of temperature & humdity on population dynamics of insects’ pest complex of cotton crop" was retracted in 2022. Reasons: compromised peer review; a conflict of interest; concerns about the authorship.

# Effect of temperature & humdity on population dynamics of insects’ pest complex of cotton crop

**DOI:** 10.1371/journal.pone.0263260

**Published:** 2022-05-06

**Authors:** Muhammad Amjad Bashir, Munaza Batool, Huma Khan, Muhammad Shahid Nisar, Hasnain Farooq, Mohamed Hashem, Saad Alamri, Manal A. El-Zohri, Reem A. Alajmi, Muhammad Tahir, Rashid Jawad

**Affiliations:** 1 Department of Plant Protection, Faculty of Agricultural Sciences, Ghazi University, Dera Ghazi Khan, Punjab, Pakistan; 2 Department of Soil & Environmental Sciences, Faculty of Agricultural Sciences, Ghazi University, Dera Ghazi Khan, Punjab, Pakistan; 3 Medical Officer Health Department Government of Punjab, BHU, Thatta Gabolan, Kot Chutta, Dera Ghazi Khan, Punjab, Pakistan; 4 Department of Environmental Sciences, University of California, Riverside, CA, United States of America; 5 Department of Forestry, Faculty of Agricultural Sciences, Ghazi University, Dera Ghazi Khan, Pakistan; 6 Botany and Microbiology Department, Faculty of Science, Assiut University, Assiut, Egypt; 7 Zoology Department, College of Science, King Saud University, Riyadh, Saudi Arabia; 8 Department of Horticulture, Faculty of Agricultural Sciences, Ghazi University, Dera Ghazi Khan, Punjab, Pakistan; Anhui Agricultural University, CHINA

## Abstract

The current study was directed to investigate the effect of temperature and humidity on insect pest complex of cotton. This study was carried out on the farmer field of a farmer of MouzaMehraywala tehsil and district Rajanpur southern part of the Punjab, Pakistan (29.1044° N, 70.3301° E) in the month of May, 2019 to November 2019. The climatic conditions of the study site were; a Rajanpur lie on 96m above sea level Rajanpur has a desert climate. During the year, there is virtually no rainfall. The average temperature in Rajanpur is 26.0°C | 78.8°F. Precipitation here is about 205 mm / 8.1 inch per year. Our results indicate that’s the correlation of temperature (minimum and maximum), humidity (minimum and maximum), rainfall and weather condition (clear or cloud), it is clear that except temperature there is a positive correlation of jassid population. While among the relation of jassid with different factor there is very weak relation with jassid population regarding temperature (-0.001), the relation of humidity, rainfall and sky condition with jassid population is positive and moderate (0.520, 0.668 & 0.575 respectively), while the relation of jassid population among these factor is significant except temperature. The results indicate that’s the correlation of temperature, humidity, rainfall and weather condition, it is clear that there is positive correlation of thrips population. While among the relation of thrips with different factor there is very weak relation of thrips population with temperature (.103), the relation of humidity, rainfall and sky condition with thrips population is positive and moderate (.515.751& .577 respectively), while the relation thrips population among these factor is significant except temperature. The results indicate that’s correlation of temperature, humidity, rainfall and weather condition, it is clear that there is positive correlation of Whitefly population. While among the relation of Whitefly with different factors there is very moderate relation of Whitefly population with temperature (.076), the relation of humidity, rainfall and sky condition with Whitefly population is negative and moderate (-.051.-.368 & -.559 respectively), while the relation Whitefly population among these factor is significant except temperature.

## Introduction

Pakistan is an agricultural country with an annual Gross Domestic Production (GDP) of about 21 percent from agricultural sector. Cotton has a pivotal position in the country agro-based economy. It is top listed cash crop of the country, which besides earning a substantial foreign exchange provides bread and butter to the millions of people from field to factories. It contributes respectively about 7 and 10 percent to agricultural value-added and GDP of the country [1]. During the growing time of cotton, however, a number of sucking and chewing insect / mite species are likely to be attacked in the field, causing significant decrease both in yield quantity and quality [2]. In Indo-Pak climate, American cotton region, G. Sweeping insect / mite pests and boltwortem complex are more likely to strike than desi cotton hirsutum (L.) [3].

Cotton is a natural fibre of great economic importance as a raw material for cloth; and is predominantly cultivated in most of the cotton producing countries of the world including Pakistan [4]. During the year 2011–12, the world total cotton production was 26.96 million tons, and China remained the main contributing country with production of 7.40 million tons, followed by India, USA, Pakistan and Brazil with production of 5.69, 3.39, 2.35 and 2.00 million tons, respectively. The area under cotton cultivation in Pakistan during the year 2011–12 was 2835 thousand hectares showing 5.4 percent increase over 2010–12; while the total cotton production in the country was 13595 thousand bales showing a tremendous increase of 18.6 percent over the preceding year. The average seed cotton yield during the year 2011–12 was 815 kg per hectare showing an increase of 12.6 percent over the yield of 724 kg per hectare during the year 2010–11 [5].

It has been well established that insect pests are major factors constraining achievement of yield potentials in Pakistan [6]. The major insect pests of cotton such as thrips, *Thripstabaci* (Lind.); jassid, *Amrascadevastans* (Dist.); whitefly, *Bemisiatabaci* (Genn.); aphid, *Aphis gossypii* (Glav.); mite, *Tetranychuscinnabarinus* (Boise); spotted bollworm, *Eariasinsulana* (Boise); pink bollworm, *Pectinophoragossypiella* (Saund) and American bollworm, *Helicoverpaarmigera* (Hub.) [7]. The insect pest infestation cause deterioration in lint quality and 10–40% losses in crop production have been noted [8].

Cotton is one of the oldest cultivable groups to be used for at least 7000 years as fibre raw material *(Gossypium spp*. tribe of Gossypieae, Malvaceae family). It is herb of more than 50 species found in arid or semi-arid tropical and subtropical regions, one of the most valuable fibre and cash crop in Pakistan. The cotton field was 3054,000 hectare in 2007 and 11,655,000 cottons were harvested [9]. Pakistan has gone from 1992 to 2000 by growing yields to 641 kilogrammes per hectare.

Among a number of low yield causes is the degree of insect pests that affect cotton from seed to maturity. Insect pests cause average losses of 5–10% but severe attacks by insect pests can lead to severe qualitative losses and losses of between 40% and 50%. Varietal resistance without use of insecticide is enormous without different tactics in the pest control [10].

Cotton insect pest complex is divided into two categories of insect pest swallowing and insect pest chewing. The most important insect sucking plagues are Whitefly and Jassid (*A*.*biguttula*). They are also known as primary pesticides causing much of the cotton damage (*T*.*tabaci*) and *A*.*gossypii*. Cotton white fly kills the plant with the sucking of a leaf curl virus vector that affects our cotton industry. It serves as the primary host of over 100 crop viruses, leading many commercial crops in various areas of the world to develop diseases [11].

Heavy infestations can reduce the vigour and growth of plants, causing chlorosis and uneven bollards. The direct feeding leads to physiological disorders which lead to the removal of immortal fruiting elements. The nymphs develop black sooty wax, which limits the photosynthesis of plants. Likewise, Jassid is also a popular cotton plant insect pest [3]. The most harmful of these are insect vector sucking complexes (*B*.*tabaci*, Homoptera: Aleyrodidae), jassid (*A*. *devastans*, Homoptera: Cicadellidae), thrip (*T*.*tabaci*,Thysanoptera: Thripidae) [12].

These sucking pests of insect / mite cause incremental delays in the vigour of the plant and the deterioration in the quality and quantity of the cotton lint [13]. Whitefly was listed for the last few years as the most significant cotton bug. Not only does this insect pest break away from the host plant but it also encourages the spread of the cotton leaf curl virus among cotton plants [14, 15]. In the cotton field in the entire world, thrips, thrips and spiders seriously infest cotton plants apart from whitespan and jassid, and decrease cotton yield and fibre quality. Insect threats such as the Thrips and the whitefly are a significant threat to cotton production in the world as a result of sucking *(B*.*tabaci*(Genus) and the jassid (*A*.*biguttula*) Quality, quantity and yield of cotton are decreased due to severe attacks by sucking insect pests. Jassid is the main threat for worldwide cotton growers, including Pakistan, among the sucking insect pests [16].

The cotton whitefly (*B*.*tabaci*Genn.) is responsible for serious economic damage in cotton crops due to Jassid infestations. When cotton is polluted with whitefly honeydew, yield quality and marketability are diminished. The lack of yield comes from feeding, and in addition, pathogenic viruses can be spread. Given the costly, environmentally destructive and highly inefficient chemical controls on this pesticide, advanced pest control software is being created. One portion of the programme is for the production of whitefly resistant cotton cultivars. Two morphological features of cotton leaves, i.e. the width of the leaves’ sinus and the density of the leaves’ fur, have been studied [17].

Jassid are distributed worldwide, but are most common in temperate zones. In contrast to many taxa. All species diversity is much lower in the tropics than in the temperate zones [18]. They can migrate great distances, mainly through passive dispersal by winds. Jassidmay also rise up in the day as high as 600 m where they are transported by strong winds [19].

The stages of life of aphids vary and have different polymorphic patterns. Aphids may be classified into heteroic (hostalternative) and monoecious (non-hostalternating) groups by their associations with host plants, which are expressed in the phenology of aphid communities, i.e. in the particular temporal cycles within one year of the flight operations, or throughout the growing season as in farm ecosystems. The seasonal flight behaviour patterns of host alternating species can be regarded as the optimum host transportation time between primary (mainly woody) and secondary (grass) hosts [20]. In non hostalternating species, seasonal flight patterns are Aphid phenology is, however, primarily determined by local environmental influences such as photoperiod and mean winter temperatures » 3 «, as well as by unique relationships between the aphid and the host plant. Climate conditions that affect aphid phenology differ and are difficult to forecast during the growing season. More complexity is added because not only inherent phenology, but also aphid abundance relies on the timing of the trap capture [21].

The populations of white and jassid typically associate positive with the temperature when the relative humidity is low. In excessive use of insecticides, resistance to these pests has not only been induced, but the climate and other health risks have also been poisoned [22]. In order to establish a strategy for the management of pests it is important to consider the nature of host selection and the influence of different morphological plants. Amrascabiguttula, Cotton Jassid, is one of India’s most significant cotton sucking pests causing a 20% reduction in yield [23]. Nymphs and adults suck the sapphire from the base of the stems, allowing the leaf to roll back, to yellow and to redden, resulting later in hopper burns and extreme pain. Pest is also a significant contributor to farmers’ growth the details about pesticide occurrence in the harvest season [24].

Pesticides used for whitefly protection typically contain active ingredients such as clothianidin, over-sell and natural, imidacloprid and thiamethoxam as well as generic additives. If swallowed, neonicotinoids may be harmfuL. Insect selection from different families may help to prevent pesticide tolerance. The same families are clothianidine and dinotefuran. Another area is treating leaves with insecticide soap [25]. The population of *B*. *tabaci* had a significant impact when the temperature changed. High temperature resulted in a decrease in the pest population. This is possibly due to the fact that the immature stages of *B*. *tabaci* were desiccated when the temperature high. Relative humidity, both high and low, were unfavorable conditions for the survival of immature stages of *B*. *tabaci* [26].

Climate conditions, for example ambient air temperature; relative humidity and rainfall, significantly influence the occurrence of pests. Both the production yield and consistency of cotton are considerably diminished by insect pests. All insect pesticides are very dependent on their effect and growth, including temperature, relative humidity and precipitation, on the predominant environmental factors. American cotton is more vulnerable to sucking pests and bollworm complexes than desi cotton (*G*. *arborium*) [27]. In addition, the growth, incidence and population modification of insect pests throughout the cotton season is determined by other weather parameters such as rainfall and temperatures, and humidity. Weather parameters such as moisture and temperature also alter the population of the jassids. The jassid populations have a significant positive temperature correlation.

Temperature is one of the most critical environmental factors influencing rate of insect growth and development. Developmental rate is usually used to quantify the effect of temperature. Previous studies have shown that temperature regulates seasonal and daily cycles, and thus indirectly influences various aspects of insect biology, such as sex ratio, adult life span, survival, fecundity, and fertility [28]. As a result, temperature profoundly affects colonization, distribution, abundance, behavior, life history, and fitness of insects [29]. Therefore, information on the thermal requirements of intrusive insect pests’ development has important implications for control programs, as temperature determines the population growth and size of intrusive pests and their variation under different conditions [30].

## Materials and methods

### Study site

This study was carried out on the farmer field of a farmer of MouzaMehraywala tehsil and district Rajanpur southern part of the Punjab, Pakistan (29.1044° N, 70.3301° E) in the month of May, 2019 to November 2019. The climatic conditions of the study site were; a Rajanpur lie on 96m above sea level Rajanpur has a desert climate. During the year, there is virtually no rainfall. The average temperature in Rajanpur is 26.0°C | 78.8°F. Precipitation here is about 205 mm | 8.1 inch per year.

### Name of variety

Variety name was BS-15. A good variety of cotton which is maximum use in south Punjab.

All the cotton was sowing at 15/05 /2019.

### Data collection

Insect pest population data were collected from the disease screening field sown. For sucking pests ten plants were selected. Sucking pests’ numbers from upper, middle and lower leaf of selected plants were counted and calculated on weekly basis. Differences were estimated on the basis of mean population. The data of different environmental factors such as maximum and minimum temperature, relative humidity during (RH) the growth period of the crop was acquired from the website www.uaf.edu.pk.

#### Method

Data regarding insect pest complex were recorded on per leaf basis observations were made early in the morning between 7:00 to 10:00 am at weekly intervals. Data was taken on 5 randomly selected plants, taking two leaves from top of the first plant, two leaves from the middle portion of the second and two from bottom portion of the next plant in each replication of each treatment. Meteorological data regarding mean daily temperature, relative humidity and rainfall were acquired from the meteorological observatory of plant physiology.

### Data analysis

The data collected were subjected to statistical analysis using State regression and correlation. SPSS Associations between insect pest populations and cotton genotypes, as well as, weather factors were estimated. The results are graphically depicted to determine the comparative response of genotypes to insect pests and to see the effect of different weather parameters on the incidence and development of insect pests.

## Results

The results indicate the correlation of temperature (minimum and maximum), humidity (minimum and maximum), rainfall and weather condition (clear or cloud). While among the relation of insects with different factor with temperature, the relation of humidity, rainfall and sky condition with insect’s population is positive, negative and moderate while the relation of insect population among all these factor.

For results we have find out the correlation of temperature (minimum and maximum), humidity (minimum and maximum), rainfall and weather condition (clear or cloud), it is clear that except temperature there is a positive correlation of jassid population (Fig 1). While among the relation of jassid with different factor there is very weak relation of jassid population with temperature (-0.001), the relation of humidity, rainfall and sky condition with jassid population is positive and moderate (0.520, 0.668 & 0.575 respectively), while the relation of jassid population among these factor is significant except temperature.

**Fig 1:** Correlation of temperature (minimum and maximum), humidity (minimum and maximum) and rainfall.

For results we have find out the correlation of temperature (minimum and maximum), humidity (minimum and maximum), rainfall and weather condition (clear or cloud), from the Fig 2, it is clear that there is positive correlation of thrips population. While among the relation of thrips with different factor there is very weak relation of thrips population with temperature (.103), the relation of humidity, rainfall and sky condition with thrips population is positive and moderate (.515.751& .577respectively), while the relation thrips population among these factor is significant except temperature (Fig 2).

**Fig 2:** Correlation of temperature (minimum and maximum), humidity (minimum and maximum) and rainfall.

For results we have find out the correlation of temperature (minimum and maximum), humidity (minimum and maximum), rainfall and weather condition (clear or cloud), from the Fig 3, it is clear that there is positive correlation of Whitefly population. While among the relation of Whitefly with different factor there is very moderate relation of Whitefly population with temperature (.076), the relation of humidity, rainfall and sky condition with Whitefly population is negative and moderate (-.051.-.368 &-.559 respectively), while the relation Whitefly population among these factor is significant except temperature (Fig 3).

**Fig 3:** Correlation of temperature (minimum and maximum), humidity (minimum and maximum) and rainfall.

For results we have find out the correlation of temperature (minimum and maximum), humidity (minimum and maximum), rainfall and weather condition (clear or cloud), from the Fig 4, it is clear that there is positive correlation of Mealy Bug population. While among the relation of Mealy Bug with different factor there is very strong relation of Bug population with temperature (-.095), the relation of humidity, rainfall and sky condition with Mealy Bug population is negative and moderate (-.074.-756-.792 &respectively), while the relation Bug population among these factor is significant except temperature (Fig 4).

**Fig 4:** Correlation of temperature (minimum and maximum), humidity (minimum and maximum) and rainfall.

For results we have find out the correlation of temperature (minimum and maximum), humidity (minimum and maximum), rainfall and weather condition (clear or cloud), from the Fig 5, it is clear that there is positive correlation of American population. While among the relation of American with different factor there is very strong relation of American population with temperature (-.036), the relation of humidity, rainfall and sky condition with American population is negative and moderate (—.313.-. 0.382. 276 & respectively), while the relation American population among these factor is significant except temperature (Fig 5).

**Fig 5:** Correlation of temperature (minimum and maximum), humidity (minimum and maximum) and rainfall.

For results we have find out the correlation of temperature (minimum and maximum), humidity (minimum and maximum), rainfall and weather condition (clear or cloud), from the Fig 6, it is clear that there is very weak relation of Armyworm population with temperature (-.119 the relation of humidity, rainfall and sky condition with Armyworm population is negative and moderate (-.024, -.518, -.492 & respectively), while the relation Armyworm population among these factor is significant except temperature (Fig 6).

**Fig 6:** Correlation of temperature (minimum and maximum), humidity (minimum and maximum) and rainfall.

For results we have find out the correlation of temperature (minimum and maximum), humidity (minimum and maximum), rainfall and weather condition (clear or cloud), from the Fig 7, it is clear that there is positive correlation of Armyworm population. While among the relation of Armyworm with different factor there is very weak relation of Armyworm population with temperature (-.119 the relation of humidity, rainfall and sky condition with Armyworm population is negative and moderate (-.024, -.518, -.492 & respectively), while the relation Armyworm population among these factor is significant except temperature (Fig 7).

**Fig 7:** Correlation of temperature (minimum and maximum), humidity (minimum and maximum), and rainfall.

For results we have find out the correlation of temperature (minimum and maximum), humidity (minimum and maximum), rainfall and weather condition (clear or cloud), from the Fig 8, it is clear that there is positive correlation of Pink boll worm population. While among the relation of Armyworm with different factor there is very weak relation of Pink boll worm population with temperature .261 the relation of humidity, rainfall and sky condition with Pink boll worm population is negative and moderate (-.086, -.122, -.278& respectively), while the relation Pink boll worm population among these factor is significant except temperature (Fig 8).

**Fig 8:** Correlation of temperature (minimum and maximum), humidity (minimum and maximum), and rainfall.

## Discussion

The current study was design to find out the effect of temperature and humidity on insect pest complex of cotton. This study was carried out on the farmer field of a farmer of MouzaMehrayWalatehsil and district Rajanpur southern part of the Punjab, Pakistan (29.1044° N, 70.3301° E) in the month of May, 2019 to November 2019. The climatic conditions of the study site were; a Rajanpur lie on 96m above sea level Rajanpur has a desert climate. During the year, there is virtually no rainfall. The average temperature in Rajanpur is 26.0°C | 78.8°F. Precipitation here is about 205 mm | 8.1 inch per year. Variety name was BS-15. A good variety of cotton which is maximum use in south Punjab. All the cotton was sowing on dated May 15, 2019.

Our results indicate that’s the era is a correlation of temperature (minimum and maximum), humidity (minimum and maximum), rainfall and weather condition (clear or cloud).it is clear that except temperature there is a positive correlation of jassid population. While among the relation of jassid with different factor there is very weak relation of jassid population with temperature, the relation of humidity, rainfall and sky condition with jassid population is positive and moderate, while the relation of jassid population among these factors is significant except temperature. Our results were approximately similar to [31].

According to [32] evaluated the studies on seasonal abundance the mean population of jassids. Incidence of the jassids and whitefly were started in 31 standard weeks with 0.4/cage and 0.2/cage, respectively. The jassids population had significant positive correlation with sunshine and evaporation and non-significant with other factors.

In our all over results we find that’s the correlation of temperature (minimum and maximum), humidity (minimum and maximum), rainfall and weather condition (clear or cloud). it is clear that there is positive correlation of thrips population. While among the relation of thrips with different factor there is very weak relation of thrips population with temperature (.103), the relation of humidity, rainfall and sky condition with thrips population is positive and moderate, while the relation thrips population among these factors is significant except temperature [33]. The data on correlation between meteorological factors and thrips population revealed that the population exhibited a positive correlation with maximum temperature while the correlation was negative with minimum and mean temperature, maximum, minimum and mean relative humidity and average rainfall. The findings confirmed the results obtained by [30] who reported negative correlation between thrips population, rainfall and temperature, similar results were also obtained by [34] who observed that the activity of thrips on different plants.

As our results the correlation of temperature (minimum and maximum), humidity (minimum and maximum), rainfall and weather condition (clear or cloud). It is clear that there is positive correlation of Whitefly population. While among the relation of Whitefly with different factor there is very moderate relation of Whitefly population with temperature, the relation of humidity, rainfall and sky condition with Whitefly population is negative and moderate, while the relation Whitefly population among these factors is significant except temperature. While our results are same as the results of Relative Humidity had significant influence on *B*. *tabaci* population and linear regression model explained 78to 85% variability in *B*. *tabaci* population development. There was negative correlation *i*.*e*. as the Relative Humidity increased the *B*. *tabaci* population decreased. The maximum influence of Relative Humidity was observed in the case of big beef where it contributed 85% towards *B*. *tabaci* population development. Rainfall had no significant influence on *B*. *tabaci* population and polynomial regression explained 35 to 42% of the variability in *B*. *tabaci* population development. The rainfall explained 42% variability in *B*. *tabaci* population. The whitefly, *B*.*tabaci*(Genn.) appeared in the third week of July (29th meteorological week) and continue up to fourth week of November (48th meteorological week) [35]. The population increased gradually and touched its peak with mean population of 6.9 whiteflies / 3leaves /plant in first week of September (36th meteorological week) during 2006–07 while, the population of whitefly touched its peak with whiteflies. The population exhibited positive correlation with maximum, minimum and mean temperature, maximum, minimum and mean relative humidity during both the study years [36]). The findings confirmed with the results obtained by [37].

For results we have find out the correlation of temperature (minimum and maximum), humidity (minimum and maximum), rainfall and weather condition (clear or cloud. it is clear that there is positive correlation of Mealy Bug population. While among the relation of Mealy Bug with different factor there is very strong relation of Bug population with temperature, the relation of humidity, rainfall and sky condition with Mealy Bug population is negative and moderate, while the relation Bug population among these factor is significant except temperature. For results we have find out the correlation of temperature (minimum and maximum), humidity (minimum and maximum), rainfall and weather condition (clear or cloud). it is clear that there is For results we have find out the correlation of temperature (minimum and maximum), humidity (minimum and maximum), rainfall and weather condition (clear or cloud),.-8, it is clear that there is positive correlation of Pink boll worm population. While among the relation of Armyworm with different factor there is very weak relation of Pink boll worm population with temperature .261 the relation of humidity, rainfall and sky condition with Pink boll worm population is negative and moderate, while the relation Pink boll worm population among these factor is significant except temperature [38–40].

The results indicate that’s correlation of temperature (minimum and maximum), humidity (minimum and maximum), rainfall and weather condition (clear or cloud). It is clear that there is positive correlation of Armyworm population. While among the relation of Armyworm with different factor there is very weak relation of Armyworm population with temperature (-.119 the relation of humidity, rainfall and sky condition with Armyworm population is negative and moderate (-.024, -.518, -.492 & respectively), while the relation Armyworm population among these factor is significant except temperature. Our results like as [41]. The population dynamics and key mortality factors of the Oriental armyworm, *Mythimnaseparata* (Walker) (Lepidoptera: Noctuidae), a serious pest of cereal crops in Asia and Australia, were studied in southern India. Adults were generally caught in light traps 15–20 days after the initiation of the monsoon rains in the first week of June, and reached a peak in September, nearly one month after the peak in larval density. Rainfall and maximum and minimum relative humidity were positively associated moth catches in the light traps [42].

## Conclusion

From above findings we concluded that correlation of temperature (minimum and maximum), humidity (minimum and maximum), rainfall and weather condition (clear or cloud) have a good effect on insect pest complex of cotton.

## Supporting information

S1 Data (XLSX)
